# Self-Expandable Metal Stent as a Bridge to Surgery for Left-Sided Acute Malignant Colorectal Obstruction: Optimal Timing for Elective Surgery

This article has been retracted.

**DOI:** 10.1155/2022/6015729

**Published:** 2022-08-16

**Authors:** Shuxian Chen, Sisi Zhou, Yiting Lin, Wenwen Xue, Zeyu Huang, Jing Yu, Zefeng Yu, Suzuan Chen

**Affiliations:** Department of Digestive Disease, First Affiliated Hospital of Shantou University Medical College, Guangdong Province 515061, China

## Abstract

**Objectives:**

This randomized, single-center, retrospective, comparative cohort study is aimed at investigating the optimal time interval from self-expandable metal stent (SEMS) placement to surgery and potential risk factors for complications in patients with acute malignant colorectal obstruction.

**Methods:**

A total of 64 patients with left-sided acute malignant colorectal obstruction treated with SEMS placement and subsequent surgery between January 2013 and September 2020 were enrolled and allocated to a case group (SEMS placing time ≤ 14 days; *n* = 19 patients) and a control group (SEMS placing time > 14 days; *n* = 45 patients). The primary outcome was the difference in baseline information, patients' conditions during surgery, and postoperative conditions between the two groups. The secondary outcome included potential risk factors of postoperative complications. The propensity score matching (PSM) and super learner (SL) methods were used to eliminate multiple confounding factors of baseline data. A cohort of 21 samples was used for external validation, comprising 6 cases and 15 controls.

**Results:**

A significant difference was observed between the two groups in intraoperative blood loss (*P* = 0.009), postoperative hospital stay (*P* = 0.002), postoperative complications (Clavien-Dindo grading ≥ II) (*P* < 0.001), stoma creation (*P* < 0.001), and primary anastomosis (*P* < 0.001). After a 1 : 3 PSM analysis, no statistically significant differences between eight confounding variables of the two groups were observed (*P* > 0.05). Caliper set as 0.2 multiple logistic regression analysis showed that the potential risk factor for postoperative complications was SEMS placing time (RR = 0.109, 95% confidence interval (CI) = 0.028-0.433; *P* = 0.002), indicating that SEMS placing time > 14 days was an independent risk factor for postoperative complications in bridge-to-surgery (BTS) setting. The area under the AUC curve was 76.7% and validated using the validation cohort.

**Conclusions:**

Long duration of SEMS placement (>14 days) may not influence surgical difficulty but could increase the risk of postoperative complications.

## 1. Introduction

At initial diagnosis, 8% to 29% of colorectal cancer patients present with symptoms of acute bowel obstruction [1]. Conventionally, patients with acute malignant colorectal obstruction receive emergency surgery (ES), which often results in stoma creation and is associated with a mortality rate of 15-34% and morbidity of 32-64% [2].

Self-expandable metal stents (SEMS) were first used for palliation of acute malignant colorectal obstruction in the 1990s and have been increasingly used as an alternative to ES bridge to surgery (BTS) [3]. The placement of SEMS before surgery could facilitate bowel decompression, stabilize patients' clinical condition, and allow for accurate tumor staging before surgery [4, 5]. Compared with ES, meta-analyses [6, 7] published in recent years have shown comparable or higher rates of primary anastomosis and lower rates of temporary colostomy and postoperative complications in the BTS group.

Despite the above benefits, the long duration of SEMS placement may increase the risk of SEMS-related complications. Among them, bowel perforation was shown to be associated with worse oncological outcomes [8, 9]. So far, there is limited data to determine the optimal interval between SEMS placement and surgery when colonic stenting is performed as BTS. A retrospective study by Matsuda et al. recommended an interval of over 15 days for minimizing postoperative complications in BTS [10]. In addition, based on low-quality evidence, a recently updated European Society of Gastrointestinal Endoscopy (ESGE) guideline recommended a time interval to surgery of approximately 2 weeks after SEMS placement when colonic stenting is performed as BTS [11].

This study is aimed at investigating the optimal time interval from SEMS placement to surgery and the risk factors for postoperative complications in patients with acute malignant colorectal obstruction.

## 2. Method

### 2.1. Patients and Study Design

Our retrospective, case-control study was approved by the Research Ethics Commission of the First Affiliated Hospital of Shantou University Medical College (2020-P-018) (Shantou, China). The requirement for informed consent was waived since this was a retrospective study.

The data of 186 patients who underwent SEMS placement at the tertiary center of the First Affiliated Hospital of Shantou University between January 2013 and September 2020 were retrieved. Those confirmed by pathology, clinical symptoms, and the endoscopic or radiologic findings (abdominal X-ray or CT) to have colorectal cancer were included. Meanwhile, patients with metastatic colorectal cancer, malignant obstruction in the right-sided colon, previous colorectal surgery, contraindications to surgery, and palliative intent were excluded. Finally, 64 patients with acute malignant left-sided colorectal obstruction undergoing SEMS placement and subsequent surgical resection were eligible and divided into a case group (SEMS placing time ≤ 14 days; *n* = 19) and a control group (SEMS placing time > 14 days; *n* = 45) following the recommendations of the European Society of Gastrointestinal Endoscopy (ESGE). In this study, the 14-day reference period refers from the day of stent placement till the day of surgical resection. In addition, a cohort including 21 patients, also divided into a case group (*n* = 6) and a control group (*n* = 15), was used as the validation dataset.  Figure 1 shows the flowchart for patient inclusion.

To minimize bias, two assistant clinical researchers unaware of the study's purpose reviewed, collected, and cross-checked the electronic medical records data, and two professional statisticians also unaware of the clinical surgery performed the statistical analyses.

### 2.2. SEMS Placement and Surgery Procedure

All patients were given enemas for bowel preparation before SEMS placement, which was performed under endoscopic and/or fluoroscopic guidance. Uncovered WallFlex (Boston Scientific, Marlborough, MA) stents, whose size, length, and diameter were selected according to the length measured at the location of the obstruction, were used. The stent was made to extend beyond the stricture at both ends by at least 2 cm. After the resolution of obstructive symptoms by SEMS placement, the patients underwent elective resection. Patients whose stent placement failed proceeded to emergency surgery.

This study defined BTS as an elective or emergency surgery after SEMS placement, independent of the time between SEMS placement and surgery. The approach and type and extent of the surgery were determined by the surgeons according to the location and stage of the primary tumor and the patient's general condition.

### 2.3. Data Description

Patients' characteristics, including baseline data (age, gender, degree of obstruction, location of tumor, SEMS placing method, American Society of Anesthesiologists score, TNM staging of tumor, and adjuvant chemotherapy), initial biochemical examination before surgery (albumin, hemoglobin), operation-related variables (surgical approach, duration of surgery, intraoperative blood loss, harvested lymph nodes, primary anastomosis, and stoma creation), and postoperative clinical variables (postoperative complications (Clavien-Dindo grading [12] ≥II), postoperative hospital stay, overall hospital stay) were collected and retrospectively reviewed.

### 2.4. Statistical Analysis

All statistical data analyses were conducted using R v3.6.3. The significance level was set at a *P* value < 0.05.

#### 2.4.1. Sample Size Calculation

The sample size calculation was performed by PASS11, as previously described [10]. The probabilities in this study to achieve a reduction in post complications were 0.0357 for SEMS placing time > 14 days and 0.368 for SEMS placing time ≤ 14 days. The trial had more than 90% power, and a two-tailed alpha of 5% was used to detect differences between the two groups with a sample size of 16 subjects with SEMS placing time ≤ 14 days and 31 subjects with SEMS placing time > 14 days.

#### 2.4.2. Difference Analysis between Two Groups

The continuous variables were presented as mean ± standard deviation (SD) or median (interquartile range (IQR): 25th-75th percentile) for continuous variables. Difference analysis was performed using Student's *t*-test or Wilcoxon signed-rank test to compare differences. The categorical data was presented as number and percentage, and differences between the two groups were analyzed using chi-square tests.

#### 2.4.3. Mining Potential Risk Factors of Postoperative Complications

Confounding variables are variables associated with both the study factor and the disease that can distort (mask or exaggerate) the true association between the factor and the disease, if unevenly distributed between the two groups compared [13]. In this study, several potential confounders, including gender, age, degree of obstruction, location of the tumor, SEMS placing method, surgical approach, preoperative albumin, preoperative hemoglobin, American Society of Anesthesiologists score, TNM staging of the tumor, harvested lymph nodes, adjuvant chemotherapy, and stoma creation, were associated with the treatment and the outcome. Accounting for these multiple potential confounders, the propensity score matching (PSM) method and super learner (SL) were adopted.

PSM randomly paired each patient in the SEMS placing time ≤ 14 days group with patients in the SEMS placing time > 14 days group based on the similarity of their propensity score [14]. Therefore, all covariates were matched to make an unbiased comparison between the groups [15] for mining potential postoperative complications risk factors. Genetic matching and 10-fold cross-validation were also used [16]. The predictor variable (*X*) was the baseline data, initial biochemical examination before surgery, and postoperative clinical variables. The response variable (*Y*) was the SEMS placing time. In addition, the distributional balance histogram and a love plot of the standardized differences of means were drawn to examine the distribution of the PSM in the original and matched groups [17].

Before matching, there were statistically significant differences between the two groups in age, surgical approach, intraoperative blood loss, and other aspects (*P* < 0.05). Considering the covariable equilibrium between the two groups after matching, the caliper value was set as 0.2. After 1 : 3 matching, 15 cases of SEMS placing time ≤ 14 days were successfully matched with 45 patients (cases) with SEMS placing time > 14 days. Then, multiple logistic regression analysis was performed to identify risk factors for postoperative complications using the training set, which was then validated in the validation dataset.

## 3. Results

### 3.1. Baseline Characteristics

From the results of demographic analysis, we found significant differences between the two groups (Table 1) in surgical approach (*P* < 0.001), intraoperative blood loss (*P* = 0.009), American Society of Anesthesiologists score (*P* = 0.041), adjuvant chemotherapy (*P* = 0.025), primary anastomosis (*P* < 0.001), postoperative complications (Clavien-Dindo grading ≥ II) (*P* < 0.001), postoperative hospital stay (*P* = 0.002, 95% CI: 1.00, 8.00), and overall hospital stay (*P* < 0.001, 95% CI: -19.00, -9.00).

### 3.2. Potential Risk Factors of Postoperative Complications

PSM analysis matched 15 patients from the case group with 45 patients from the control group. No statistically significant difference was observed for 8 confounding variables between the two groups (Table 2). The histogram of distribution balance and the love graph of standardized difference are shown in Figures 2 and 3. Subsequent multiple logistic regression analysis showed that the potential risk factor for postoperative complications was SEMS placing time (RR = 0.109, 95% CI: 0.028-0.433; *P* = 0.002), indicating that SEMS placing time (≤14 days) was a protective factor for postoperative complications. The area under the AUC curve was 76.7% under the validation data (Figure 4).

## 4. Discussion

Colorectal cancer is a multifactorial disease, the third most common cancer in males and the second most common cancer in females [18, 19]. Although the BTS strategy showed a lower incidence of postoperative complications and stoma creation compared with emergency surgery [6, 7], little is known about risk factors for postoperative complications and the optimal time for the resection of the obstructed colon.

Some studies showed that postoperative complications were associated with impaired long-term survival in patients with colorectal cancer [20–22]. In this present study, the incidence of postoperative complications after BTS strategy was 25%, similar to that previously reported [3, 6, 23, 24].

Many studies have evaluated potential factors affecting postoperative complications in patients with colorectal cancer. Kim et al. performed a retrospective study and reported that older age, higher ASA score, presence of anemia, and lower serum albumin were associated with an increased incidence of postoperative complications [25]. Zhu et al. showed that postoperative complications might be associated with tumor size and site and pathological stage in patients with rectal cancer [26]. Moreover, the surgical approach also seemed to be a risk factor for postoperative complications. A randomized clinical trial investigated the short-term outcomes of laparoscopic surgery versus open surgery in patients with colorectal cancer and reported similar rates of postoperative complications [27]. However, another randomized clinical trial [28] and a retrospective study [29] reported an increase in complication rates when patients underwent conversion from laparoscopic to open surgery. In addition, the presence of a protective stoma was reported to decrease the incidence of anastomotic leakage and mitigate the clinical consequences of leakage [30].

Matsuda et al. investigated the optimal interval between SEMS placement and subsequent surgery in a BTS setting and recommended an interval of over 15 days to minimize postoperative complications [10]. Comparatively, our study demonstrated that a shorter interval from SEMS placement to surgery (≤14 days) was an independent risk factor for lower risks of postoperative complications. The reported interval between SEMS placement and surgery varied widely from 3 to 28 days [6, 7, 30] in several meta-analyses. However, there are limited data to determine the optimal time interval for surgery following SEMS placement. Lee et al. showed a higher anastomotic leakage rate in patients with an interval < 10 days (cases, 3/15) than in patients whose surgery was delayed for 10 days or longer (cases, 0/28) [23]. Theoretically, a longer interval (>1 week) could compromise surgery by more local tumor infiltration and fibrosis [31]. However, a randomized clinical trial from China reported that patients who underwent laparoscopic surgery 10 days after SEMS placement had a significantly higher primary anastomosis rate (*P* = 0.001) and a lower conversion rate than patients 3 days after SEMS placement (*P* = 0.046) [32]. Besides, a retrospective study by Matsuda et al. reported no significant differences in duration of surgery and intraoperative blood loss between patients who underwent surgery < 15 days and ≥15 days after SEMS placement [10]. In our study, we observed no significant differences in duration of surgery between patients who underwent surgery ≤ 14 days and >14 days after SEMS placement; however, compared with patients with a ≤14-day interval, patients with a >14-day interval had less intraoperative blood loss, shorter postoperative hospital stay, lower rate of postoperative complication and stoma creation, and higher rate of primary anastomosis. We hypothesize that the possible reasons for these observations could be first, long-term intestinal patency and antibiotic treatment after SEMS placement could better restore intestinal barrier function, making it difficult for bacteria to pass through the intestinal barrier and thus reduce the risk of infection complications. Second, the improvement of intestinal wall edema and ischemia was also beneficial in modifying damaging organisms and thus reducing the occurrence of anastomotic leakage. Third, all perforations after SEMS placement in our study occurred within several days, leading to the intestinal contents penetrating into the enterocoelia, thereby increasing the risk of abdominal infection. Lastly, patients who underwent surgery > 14 days after SEMS placement comprised a higher proportion of patients who underwent laparoscopic surgery and a lower proportion of patients who had open surgery than patients with a shorter time interval, suggesting a possible implication of laparoscopic surgery in reducing the risk of trauma and improving postoperative recovery time compared with open surgery. Taken together, our findings suggest that long intervals (>14 days) between SEMS placement and surgery did not influence surgical difficulty but improved the rate of primary anastomosis and reduced the rate of stoma creation and postoperative complications.

In spite of the short-term benefits discussed above, the long duration of stent placement may have a negative influence on oncologic outcomes. Several studies have reported that air or dye insufflation, guidewire insertion, and SEMS dilation could irritate the cancer and the effect of mechanical compression of the tumor could result in cancer cell spread [4, 33, 34]. In addition, the relationship between stent-related adverse events, especially in intestinal perforation, and tumor recurrence has been the focus of attention. Some studies reported that intestinal perforation increased the risk of tumor recurrence [9, 35]. However, a retrospective study by Rodrigues et al. compared long-term outcomes of BTS and ES in patients with acute malignant colorectal obstruction and found that only surgery-related adverse events, not SEMS-related adverse events, influenced overall survival and 30-day mortality [36]. So far, there are limited data on the relationship between the duration of SEMS placement before surgery and long-term oncological outcomes. Only a retrospective study conducted by Malene et al. found that a longer interval (≥18 days) was an independent risk factor for tumor recurrence, irrespective of whether the patients had or not SEMS-related adverse events [37]. In our study, no significant differences were observed in TNM stage between the two groups. Compared with patients with the ≤14-day interval, patients with a >14-day interval had more harvested lymph nodes. Lymph node metastasis is one of the important metastatic pathways of colorectal cancer. More harvested lymph nodes are beneficial to expanding the effect of radical resection and thus reducing tumor recurrence. Besides, 5 patients developed intestinal perforation a few hours to a few days after SEMS placement, while no patient in the >14-day interval group developed intestinal perforation, suggesting that the latter could be associated with a lower likelihood of developing peritoneal implantation metastasis. Therefore, we speculate that patients with >14-day interval may have better tumor outcomes, but unfortunately, we did not follow up with these patients after discharge and were unable to obtain long-term oncologic outcome data.

There were some limitations in this study. First, this was a retrospective study conducted in a tertiary referral center, and selection bias was inevitable despite performing PSM analysis. Second, the sample size within the two groups was relatively small. Lastly, the observation of postoperative complications was limited to the short postoperative hospitalization time, and no long-term outcomes were available.

In conclusion, this study findings showed that a long duration of SEMS placement (>14 days) may not increase surgical difficulty in patients undergoing surgery using the BTS strategy but was associated with improvement in the rate of primary anastomosis and reduction in the rate of stoma creation and postoperative complications.

## Figures and Tables

**Figure 1:** A flowchart for patient inclusion.

**Figure 2:** The histogram of distribution balance for “age.”

**Figure 3:** The love graph of standardized differences.

**Figure 4:** The area under the AUC curve was 76.7% in the validation data.

**Table 1:** Comparison of characteristics between the case and control groups.

Variables	Case group (*n* = 19)	Control group (*n* = 45)	*P* value
Patient-related			
Gender (*n*[%])			0.058
Male	16 (84.21)	25 (55.56)	
Female	3 (15.79)	20 (44.44)	
Age	64.73 ± 15.66	68.27 ± 9.41	0.268
ASA score (*n*[%])			0.041
1	1 (5.26)	1 (2.22)	
2	12 (63.16)	35 (77.78)	
3	3 (15.79)	9 (20.00)	
4	3 (15.79)	0 (0.00)	
Adjuvant chemotherapy (*n*[%])			0.025
Yes	1 (5.26)	15 (33.33)	
No	18 (94.74)	30 (66.67)	
Tumor location (*n*[%])			0.116
Splenic flexure	0 (0.00)	5 (11.11)	
Descending colon	2 (10.53)	7 (15.56)	
Junction of descending colon and sigmoid	0 (0.00)	4 (8.89)	
Sigmoid	15 (78.95)	18 (40.00)	
Junction of sigmoid and rectum	1 (5.26)	3 (6.67)	
Rectum	1 (5.26)	8 (17.78)	
TNM stage (*n*[%])			0.680
I	0 (0.00)	1 (2.22)	
II	4 (21.05)	15 (33.33)	
III	8 (42.11)	17 (37.78)	
IV	7 (36.84)	12 (26.67)	
Degree of obstruction (*n*[%])			0.788
Complete	9 (47.37)	18 (40.00)	
Incomplete	10 (52.63)	27 (60.00)	
Stent placement technique (*n*[%])			0.190
Endoscopy	2 (10.53)	13 (28.89)	
Fluoroscopy	5 (26.32)	6 (13.33)	
Both	12 (63.16)	26 (57.78)	
Blood examination before surgery			
Albumin (g/L), mean ± SD	33.59 ± 3.39	32.65 ± 3.48	0.322
Hemoglobin (g/L), mean ± SD	118.37 ± 16.77	112.51 ± 12.51	0.182
Surgical approach (*n*[%])			<0.001
Laparoscopic	11 (57.89)	44 (97.78)	
Open	6 (31.58)	0 (0.00)	
Conversion	2 (10.53)	1 (2.22)	
Duration of surgery (min), median (IQR)	205.00 (174.00, 285.00)	195.00 (160.00, 225.00)	0.198
Intraoperative blood loss (10/20/30/50/100/200/300/400/600) (mL)	0/2/0/5/5/3/0/0/4	1/11/1/21/5/2/3/1/0	0.009
Harvested lymph nodes	16.19 ± 9.85	21.11 ± 9.60	0.068
Primary tumor resection (*n*[%])			
Yes	19 (100.00)	45 (0.00)	
No	0 (0.00)	0 (0.00)	
Primary anastomosis (*n*[%])			<0.001
Yes	12 (63.16)	45 (100.00)	
No	7 (36.84)	0 (0.00)	
Postoperative complications (Clavien-Dindo ≥ 2) (*n*[%])			<0.001
Yes	11 (57.89)	5 (11.11)	
No	8 (42.11)	40 (88.89)	
Postoperative hospital stay (d), median (IQR)	14.00 (9.50, 20.50)	9.00 (9.00, 11.00)	0.002
Overall hospital stay (d), median (IQR)	22.00 (19.00, 27.00)	34.00 (29.00, 43.00)	<0.001

**Table 2:** Comparison of matched cases after PSM analysis.

Variables	Case group (*n* = 15)	Control group (*n* = 45)	*P* value
Gender (*n*[%])			0.063
Male	13 (86.67)	25 (55.56)	
Female	2 (13.33)	20 (44.44)	
Age	61.87 ± 10.10	68.27 ± 9.41	0.029
ASA score (*n*[%])			0.843
1	1 (6.67)	1 (2.22)	
2	12 (80.00)	35 (77.78)	
3	3 (20.00)	9 (20.00)	
4	0 (0.00)	0 (0.00)	
Adjuvant chemotherapy (*n*[%])			0.025
Yes	0 (0.00)	15 (33.33)	
No	15 (100.00)	30 (66.67)	
Tumor location (*n*[%])			0.256
Splenic flexure	0 (0.00)	5 (11.11)	
Descending colon	2 (13.33)	7 (15.56)	
Junction of descending colon and sigmoid	0 (0.00)	4 (8.89)	
Sigmoid	11 (73.33)	18 (40.00)	
Junction of sigmoid and rectum	1 (6.67)	3 (6.67)	
Rectum	1 (6.67)	8 (17.78)	
TNM stage (*n*[%])			0.877
I	0 (0.00)	1 (2.22)	
II	4 (26.67)	15 (33.33)	
III	6 (40.00)	17 (37.78)	
IV	5 (33.33)	12 (26.67)	
Degree of obstruction (*n*[%])			0.547
Complete	8 (53.33)	18 (40.00)	
Incomplete	7 (46.67)	27 (60.00)	
Stent placement technique (*n*[%])			0.465
Endoscopy	2 (13.33)	13 (28.89)	
Fluoroscopy	2 (13.33)	6 (13.33)	
Both	11 (73.33)	26 (57.78)	
Preoperative albumin (g/L), mean ± SD	34.55 ± 2.59	32.65 ± 3.48	0.057
Preoperative hemoglobin (g/L), mean ± SD	119.60 ± 16.24	112.51 ± 12.51	0.084
Surgical approach (*n*[%])			0.001
Laparoscopic	11 (73.33)	44 (97.78)	
Open	4 (26.67)	0 (0.00)	
Conversion	0 (0.00)	1 (2.22)	
Harvested lymph nodes	13.73 ± 6.63	21.11 ± 9.60	0.008
Primary anastomosis (*n*[%])			0.003
Yes	11 (73.33)	45 (100.00)	
No	4 (26.67)	0 (0.00)	
Stoma creation (including temporary diversion)			0.015
Yes	4 (26.67)	1 (2.22)	
No	11 (73.33)	44 (97.78)	

## Data Availability

The data used to support the findings of this study are available from the corresponding author upon request.
